This article has been retracted.

# Resveratrol attenuates mechanical compression-induced nucleus pulposus cell apoptosis through regulating the ERK1/2 signaling pathway in a disc organ culture

**DOI:** 10.1042/BSR20171703

**Published:** 2018-03-09

**Authors:** Zhiwen Zhang, Feng Wen, Chengjian He, Jun Yu

**Affiliations:** 1 Department of Orthopedic Surgery, Hubei Provincial Hospital of Traditional Chinese Medicine, Wuhan 430061, China; 2 Hubei Province Academy of Traditional Chinese Medicine, Wuhan 430070, Hubei, China; 3 Xiaogan No.1 People’s Hospital, Xiaogan, Hubei 432100, China

**Keywords:** apoptosis, intervertebral disc degeneration, nucleus pulposus, resveratrol

## Abstract

Background: Nucleus pulposus (NP) cell apoptosis is a typical feature within the degenerative disc. High magnitude compression significantly promotes NP cell apoptosis. Several studies have indicated that resveratrol has protective effects on disc cell’s normal biology.

Objective: The present study aims to investigate whether resveratrol can attenuate mechanical overloading-induced NP cell apoptosis in a disc organ culture.

Methods: Isolated porcine discs were cultured in culture chambers of a mechanically active perfusion bioreactor and subjected to a relatively high magnitude compression (1.3 MPa at a frequency of 1.0 Hz for 2 h once per day) for 7 days. Different concentrations (50 and 100 μM) of resveratrol were added into the culture medium to observe the protective effects of resveratrol against NP cell apoptosis under mechanical compression. The noncompressed discs were used as controls.

Results: Similar with the previous studies, this high magnitude compression significantly promoted NP cell apoptosis, reflected by the increased number of terminal deoxynucleotidyl transferase dUTP nick-end labeling (TUNEL) staining-positive NP cells and enzyme (caspase-9 and caspase-3) activity, the up-regulated expression of proapoptotic molecules (Bax and caspase-3/cleaved caspase-3), and down-regulated expression of antiapoptotic molecule (Bcl-2). However, resveratrol partly attenuated NP cell apoptosis under this high magnitude compression in a dose-dependent manner. Additionally, though the ERK1/2 pathway was significantly activated in the mechanical compression group, resveratrol partly attenuated activation of the ERK1/2 pathway under mechanical compression in a dose-dependent manner.

Conclusion: Resveratrol attenuates mechanical overloading-induced NP cell apoptosis in a dose-dependent manner, and inhibiting activation of the ERK1/2 pathway may be one potential mechanism behind this regulatory process.

## Introduction

Intervertebral disc degeneration (IDD) is a leading cause of low back and leg pain, which imposes serious socioeconomic loss and affects patient life quality [1]. Though numerous clinical and basic researches have been carried out during the past years, the potential mechanism behind IDD remains unclear. More studies are needed to develop pertinent treatments for disc degeneration.

The peripheral annulus fibrosus (AF), the central nucleus pulpous (NP), and the cartilage endplate (CEP) make up the intact intervertebral disc (IVD) [2]. During disc degeneration, the NP region first exhibits degenerative pathological changes, including decrease in normal matrix content and increase in cell apoptosis [3,4]. It is well established that cell apoptosis is one of the main causes of cell loss and that cellular loss from NP cell apoptosis indeed contributes to disc degeneration [5,6].

As a load absorbing structure of spine, the IVD is subjected to various modes and magnitudes of mechanical compression during the daily life. Previously, numerous studies have demonstrated that mechanical compression plays a crucial role in regulating disc cell viability and biosynthetic function [7–9]. Moreover, high magnitude compression significantly promotes disc degeneration [10]. Importantly, a previous study has demonstrated that high magnitude compression significantly promotes NP cell apoptosis in NP cell–scaffold culture system and in the intact disc organ culture system [11]. Based on the above statements, we speculate that attenuation of NP cell apoptosis may be an effective strategy to attenuate high magnitude compression-induced disc degeneration.

Resveratrol is a natural phytoalexin found in plants including peanuts and grapes [12]. Recently, resveratrol is reported to have wide protective effects in different cell types, such as the anti-inflammatory, antiaging, and cartilage protection [13–15]. Therefore, in the present study, we mainly aimed to investigate whether the resveratrol can attenuate mechanical compression-induced NP cell apoptosis and the subsequent alteration of ERK1/2 pathway activity in this regulatory process.

## Materials and methods

### Ethical statement

All experiments were complied with the protocol of the Ethics Committee at Hubei Provincial Hospital of Traditional Chinese Medicine [SHNK (E) 2015-0022].

### Disc isolation and bioreactor culture

Ten healthy pigs (male, 10–13 kg, 3–4 months old) were receiving standard housing and husbandry before disc harvest. The intact discs were isolated according a previous study [11]. Briefly, after experiment animals were killed via intravenous injection of an overdose of pentobarbital sodium (100 mg/kg), the spinal column was separated, and then the attached connective tissue and ligaments were removed as much as possible. Thereafter, the intact discs (Th11/Th12-L4/L5) with CEPs were isolated under a dissecting microscope. Finally, the isolated discs were rinsed with phosphate buffer solution (PBS) and perfusion-cultured for 7 days in the culture chambers of a perfusion and mechanically active bioreactor. In the meantime, the discs were experienced with a high compressive magnitude of 1.3 MPa at the frequency of 1.0 Hz for 2 h once per day. The 1.3 MPa of compressive magnitude was regarded as mechanical overloading since it has been demonstrated to significantly promote NP cell apoptosis and is a relatively high magnitude compression in a previous study [11]. On the other hand, to investigate the potential protective role of resveratrol against high magnitude compression-induced NP cell apoptosis, the compressed discs were incubated with different concentrations (50 and 100 μM) of resveratrol that were designed according to previous studies [16,17]. The unloaded discs were regarded as the controls. Hundred milliliters of fresh DMEM/F12 culture medium (Gibco, U.S.A.) supplemented with 10% (v/v) fetal bovine serum (FBS, Gibco, U.S.A.), 1% (v/v) penicillin–streptomycin (Gibco, U.S.A.), 0.025 mg/ml ascorbic acid (Sigma, U.S.A.), and 15 mM HEPES (Sigma, U.S.A.) was circulated at a rate of 5 ml/min [18].

### Terminal deoxynucleotidyl transferase dUTP nick-end labeling (TUNEL) assay

Briefly, after the culture, discs were rinsed with PBS. Then, they were fixed with 4% paraformaldehyde, decalcified with 10% ethylenediaminetetraacetic acid (EDTA), and embedded in paraffin. After 5 μm thick cross-sections were prepared, they were dewaxed with xylene and permeated with proteinase K, TUNEL staining assay was performed according to the manufacturer’s instructions (Roche, Switzerland). Apoptotic NP cells were observed under a light microscope and quantified with the Image-Pro Plus software (Version 5.1, Media Cybernetics, Inc.).

### Caspase enzyme activity measurement

Because caspase-9 and caspase-3 are two pivotal enzymes in the mitochondria-mediated cell apoptosis [19], their activity was measured with the commercial caspase-3 and caspase-9 activity detection kit (Beyotime, China). Briefly, after disc culture, the central gelatinous NP samples were incubated with 300 μl of lysis buffer for 10 min. Then, the protein supernatant was separated by centrifugation at 15 × 10^3^ g for 15 min at 4°C. Thereafter, the reaction system containing 40 μl of buffer, 50 μl of lysate, and 10 μl of Ac-LEHD-*p*NA (for caspase-9 activity measurement), and 10 μl of Ac-DEVD-pNA (for caspase-9 activity measurement) was incubated for 8 h at 37°C. Finally, caspase-9 and caspase-3 activity were calculated by measuring the absorbance value at a wavelength of 405 nm.

### Real-time PCR analysis

Gene expression of apoptosis-related molecules (Bcl-2, Bax, and caspase-3) was analyzed by real-time PCR analysis. Briefly, total RNA was extracted from the isolated NP samples using the Tripure Isolation Reagent (Roche, Switzerland) and reverse-transcripted into cDNA using a First Strand cDNA Synthesis Kit (Roche, Switzerland). Then, the total 20 μl volume of reaction mixture containing 10 μl of SYBR Green Mix (TOYOBO, Japan), 8 μl of RNase-free water, 1.5 μl of cDNA, and 1 μl of primer mix was subjected to a real-time PCR machine (CFX96 Real-Time System, Bio-Rad). The PCR was finished according to the below parameters: 5 min at 95°C, followed by 40 amplification cycles of 25 s at 95°C, 15 s at 56°C, and 15 s at 72°C. Primers (Table 1) for each target gene were synthesized by a domestic commercial company (Sangon, Biotech Co., Ltd., China). GAPDH was used as an internal control for normalization, and the relative gene expression was calculated according to the 2^―ΔΔ*C*^_t_ method.

**Table 1:** Primers of target genes

Gene	Accession number	Forward (5′-3′)	Reverse (5′-3′)
GAPDH	NM_001082253.1	GACCACTTTGTGAAGCTCATTTC	GTGGTTTGAGGGCTCTTACTC
Bcl-2	XM_003121700.3	GGGAGGATTGTGGCCTTCTT	GGCCCATACAGCTCCACAAA
Bax	XM_003355975.2	TTCATCCAGGATCGAGCAGG	TCCAATGCGCTTGAGACACT
Caspase-3	NM_214131.1	GGGATTGAGACGGACAGTGG	TGAACCAGGATCCGTCCTTTG

### Western blotting assay

Briefly, the central NP samples were isolated under a dissecting microscope after disc bioreactor culture. Then, total protein was extracted from the isolated NP tissue using the RIPA lysis buffer (Beyotime, China). After the protein concentration was determined with a BCA kit (Beyotime, China), equal protein sample in each group was subjected to the SDS/PAGE system and transferred to the PVDF membrane. Then, incubation of primary antibodies against Bcl-2 (Proteintech, 60178-1-Ig, diluted 1:1000), Bax (Abcam, ab104156), cleaved caspase-3 (Santa Cruz, sc-7148), p-ERK1/2 (Santa Cruz, sc-101761), ERK1/2 (Santa Cruz, sc-292838), and GAPDH (Abcam, ab8245) was performed at 4°C overnight, and incubation of corresponding HRP-conjugated secondary antibodies was carried out at room temperature for 2 h. After protein bands were visualized with the ECL Plus reagent (Thermo, U.S.A.), the gray value of protein bands was measured using the ImageJ software (National Institutes of Health, U.S.A.). Protein expression was normalized to the expression of GAPDH.

### Statistical analysis

All numerical data were presented as mean ± standard error of mean (SED). SPSS 17.0 software was used to analyze the statistical difference. After the homogeneity test for variance, intergroup difference was analyzed using a one-way analysis of variance (ANOVA). The *post hoc* test was performed using the LSD test. A *P*-value<0.05 was considered as a statistical difference.

## Results

### TUNEL staining assay

As shown in the Figure 1, the percentage of staining-positive NP cells in the 1.3 MPa group significantly increased compared with the control group. However, resveratrol partly decreased the number of staining-positive NP cells in the 1.3 MP group in a dose-dependent manner, further confirming that high magnitude compression promotes NP cell apoptosis and indicating that resveratrol can partly attenuate NP cell apoptosis under mechanical compression.

**Figure 1:** Nucleus pulposus (NP) cell apoptosis detected by TUNEL staining Magnification: 200×; scale = 100 μM; *n* = 3. Data are expressed as mean ± SD. *: Indicates a significant difference (*P*<0.05) between two groups. #: Indicates a significant difference (*P*<0.05) compared with the 1.3 MPa group.

### Caspase-9 and caspase-3 activity

Both caspase-9 and caspase-3 activity in this high magnitude compression group were significantly increased compared with that in the control group. However, resveratrol significantly decreased their activity under this high magnitude compression, Moreover, the high concentration of resveratrol (100 μM) decreased caspase-9 activity and caspase-3 activity even more compared with the low concentration of resveratrol (50 μM) under this high magnitude compression (Figure 2). Collectively, these results indicate that resveratrol can decrease activity of caspase enzyme that was involved in mitochondria-mediated cell apoptosis under mechanical compression in a dose-dependent manner.

**Figure 2:** Caspase enzymes activity measurement (**A**) Caspase-9 activity analysis. (**B**) Caspase-3 activity analysis. Data are expressed as mean ± SD. *: Indicates a significant difference (*P*<0.05) between two groups. #: Indicates a significant difference (*P*<0.05) compared with the 1.3 MPa group.

### Gene expression of apoptosis-related molecules

As shown in the Figure 3, this high magnitude compression significantly down-regulated mRNA expression of antiapoptotic molecule (Bcl-2) whereas up-regulated mRNA expression of proapoptotic molecules (Bax and caspase-3). However, resveratrol partly reversed the expression profile of these molecules under mechanical compression. Moreover, the discs incubated with a high resveratrol concentration (100 μM) produced higher Bcl-2 level and lower Bax and caspase-3 levels than those incubated with a low resveratrol concentration (50 μM) under this relatively high mechanical compression. These results indicate again that resveratrol can attenuate mechanical overloading-induced NP cell apoptosis in a dose-dependent manner.

**Figure 3:** Real-time PCR analysis of apoptosis-related molecules (Bcl-2, Bax, and caspase-3) Data are expressed as mean ± SD. *: Indicates a significant difference (*P*<0.05) between two groups. #: Indicates a significant difference (*P*<0.05) compared with the 1.3 MPa group.

### Protein expression of apoptosis-related molecules

Western blotting assay showed that this high magnitude compression significantly down-regulated protein expression of antiapoptotic molecule (Bcl-2) whereas up-regulated protein expression of proapoptotic molecules (Bax and cleaved caspase-3). However, resveratrol partly reversed the protein expression profile of these molecules under this mechanical compression in a dose-dependent manner (Figure 4). These results are consistent with the results of gene expression profile and further indicate that resveratrol can attenuate mechanical overloading-induced NP cell apoptosis in a dose-dependent manner.

**Figure 4:** Western blotting analysis (A) of apoptosis-related molecules (Bcl-2, Bax, and cleaved-caspase-3) and the corresponding quantification (B-D) Data are expressed as mean ± SD. *: Indicates a significant difference (*P*<0.05) between two groups. #: Indicates a significant difference (*P*<0.05) compared with the 1.3 MPa group.

### Activity of the ERK1/2 signaling pathway

Previous study has shown that activation of the ERK1/2 pathway plays an important role in mechanical load-caused alteration of NP cell biological behaviors, and that resveratrol can regulate its activity under some external stimuli. To tentatively investigate the role of the ERK1/2 pathway in this regulatory process, we analyzed the expression of p-ERK1/2 expression in each group. Results showed that ERK1/2 pathway activity in this high magnitude mechanical compression group is sharply higher than that in the control group. Similarly, resveratrol partly attenuated activation of the ERK1/2 pathway under mechanical compression in a dose-dependent manner (Figure 5). Combined with the above results, this partly implies that inhibiting the activation of the ERK1/2 pathway may be the potential signaling transduction mechanism behind the protective effects of resveratrol against mechanical overloading-induced NP cell apoptosis.

**Figure 5:** Activity of the ERK1/2 pathway measured by Western blotting assay (A) and the corresponding quantification (B) Data are expressed as mean ± SD. *: Indicates a significant difference (*P*<0.05) between two groups. #: Indicates a significant difference (*P*<0.05) compared with the 1.3 MPa group.

## Discussion

Disc degeneration is a common health problem worldwide [20,21]. Mechanical load is an implicate regulator during disc development and remodeling [10,22]. Previous studies have reached a consensus that mechanical overloading-caused NP cell apoptosis largely contributes to disc degeneration [10]. Hence, inhibition of high magnitude compression-induced NP cell apoptosis may be helpful to retard disc degeneration caused by the unphysiological/high compressive stress. In the present study, we confirmed that mechanical overloading significantly promoted NP cell apoptosis and demonstrated that resveratrol partly attenuated mechanical overloading-induced NP cell apoptosis in a dose-dependent manner. This study provides potential therapeutic effects of resveratrol on mechanical overloading-induced disc degeneration.

Disc organ culture maintains the integrity of disc structure and the interaction between cell–cell and/or cell–tissue [23]. Recently, the disc organ culture system is regarded as a superior experiment model for studying disc biology [24]. In particular, application of the perfusion bioreactor makes the present study more closer to the physiological condition [25]. Dynamic compression is one of the common mechanical patterns experienced by the discs *in vivo*. The magnitude of 1.3 MPa and frequency of 1.0 Hz used in the present study are all within the human physiological situation [26,27]. Furthermore, the 1.3 MPa has been previously proved to be a relatively high-magnitude which can promote NP cell apoptosis and inhibit NP matrix biosynthesis [11]. Therefore, the magnitude of 1.3 MPa was considered as a destructive compression in the present study. In addition, because the mitochondria-mediated cell apoptosis is the main type of cell death during the severe disc degeneration [28], the tested parameters, such as enzyme (caspase-9 and caspase-3) activity and expression of apoptosis-related molecules (Bax, Bcl-2, and caspase-3/cleaved caspase-3), were largely focused on this cell apoptosis approach.

The mechanical function of discs mainly depends on the content and organization of the NP matrix, which is synthesized and maintained by NP cells [29]. Because cell density of the NP tissue is relatively low compared with other tissues, NP cell apoptosis-caused decrease in NP cell number poses a considerable threatening challenge upon NP matrix content [6]. During the past years, NP cell apoptosis has attracted the attention of many investigators [30,31]. To develop strategies of preventing NP cell apoptosis, many *in vitro* studies were performed. For example, Sudo et al. demonstrated that caspase-3 siRNA was able to prevent the apoptosis of rabbit NP cells [32]. Another study of this research team also showed that overexpression of Bcl-2 mRNA in rat NP cells could attenuate NP cell apoptosis [33]. To completely and preferably achieve this goal, more studies need to be performed.

In the present study, we found that NP cell apoptosis, indicated by TUNEL staining and enzyme (caspase-3 and 9) activity and expression of apoptosis-related molecules (Bax, Bcl-2, and caspase-3/cleaved caspase-3), was significantly aggravated by this high magnitude compression. This is in line with previous studies and further confirming that mechanical overloading promotes disc cell death [10,11]. Resveratrol is known to have beneficial effects, including anti-inflammatory, antiaging, and antioxidative stress [12]. In the research field of disc biology, resveratrol is reported to attenuate disc cell apoptosis and increase disc matrix synthesis in the inflammatory condition [16,17]. However, few studies investigated whether it has a similar protective effects on the mechanical overloading-induced disc NP cell apoptosis. Our results showed that resveratrol partly attenuates this high magnitude mechanical compression-induced NP cell apoptosis; moreover, its protective effect against NP cell apoptosis under mechanical compression is in a dose-dependent manner, suggesting that resveratrol can attenuate mechanical overloading-induced NP cell apoptosis in a dose-dependent manner.

The mitogen-activated protein kinase (MAPK) pathways are responsible for transmitting the external stimuli to the alteration of cellular biological behaviors, and are involved in many cell bioactivities, such as cell proliferation, cell senescence, cell apoptosis, and cell biosynthesis [34]. Previously, the existence of MAPK pathways in NP cells was also identified [35]. In the present study, inhibition of the ERK1/2 pathway was positively correlated with the attenuation of NP cell apoptosis under this high magnitude compression after resveratrol was added into the disc culture medium. Furthermore, both of them were in a resveratrol concentration-dependent manner. Combined with the protective effects of resveratrol against NP cell apoptosis under this high magnitude compression, it can be deduced that inhibiting the ERK1/2 pathway may be one potential mechanism behind this regulatory process.

In conclusion, the present study confirms again that mechanical overloading can aggravate disc NP cell apoptosis. Meanwhile, the present study demonstrates that resveratrol can alleviate disc NP cell apoptosis in a dose-dependent manner under mechanical overloading, in which it may function through inhibiting the ERK1/2 pathway. Together, the present study directly provides that resveratrol supply may be a potential strategy that can alleviate the mechanical overloading-induced disc NP cell apoptosis.

## Abbreviations

CEP: cartilage endplate
IDD: intervertebral disc degeneration
IVD: intact intervertebral disc
MAPK: mitogen-activated protein kinase
NP: nucleus pulposus
PBS: phosphate buffer solution
